The article "Analgesic Effects of Dexmedetomidine Combined with Spinal and Epidural Anesthesia Nursing on Prostate Hyperplasia Patients after Transurethral Resection of Prostate by Intelligent Algorithm-Based Magnetic Resonance Imaging" was published in 2022. Journal: Comput Math Methods Med.

# Analgesic Effects of Dexmedetomidine Combined with Spinal and Epidural Anesthesia Nursing on Prostate Hyperplasia Patients after Transurethral Resection of Prostate by Intelligent Algorithm-Based Magnetic Resonance Imaging

**DOI:** 10.1155/2022/4243244

**Published:** 2022-05-21

**Authors:** Xiaoyan Zhang, Manyun Bo, Rong Zeng, Liping Zou, Yanfang He

**Affiliations:** Department of Anesthesia Surgery, Changsha Fourth Hospital, Changsha, 410006 Hunan, China

## Abstract

To analyze the investigation of the application effects of different doses of dexmedetomidine (Dex) with combined spinal and epidural anesthesia nursing on analgesia after transurethral resection of prostate (TURP) by intelligent algorithm-based magnetic resonance imaging (MRI), MRI imaging segmentation model of mask regions with convolutional neural network (Mask R-CNN) features was proposed in the research. Besides, the segmentation effects of Mask R-CNN, U-net, and V-net algorithms were compared and analyzed. Meanwhile, a total of 184 patients receiving TURP were selected as the research objects, and they were divided into A, B, C, and D groups based on random number table method, each group including 46 cases. Patients in each group were offered different doses of Dex, and visual analogue scale (VAS) and Ramsay scores of different follow-up visit time, use of other analgesics, the incidence of postoperative cystospasm, and nursing satisfaction of patients in four groups were compared. The results demonstrated that Dice similarity coefficient (DSC) value, specificity, and positive predictive value of Mask R-CNN algorithm were 0.623 ± 0.084, 98.61%, and 69.57%, respectively, all of which were higher than those of U-net and V-net algorithms. Pain VAS scores and the incidence of cystospasm at different time periods of groups B and C were both significantly lower than those of group D (*P* < 0.05). Ramsay scores of groups B and C at 8 hours, 12 hours, 24 hours, and 48 hours after the operation were all remarkably higher than those in group D (*P* < 0.05). Besides, nursing satisfaction of groups B and C was obviously superior to that in group D, and the difference demonstrated statistical meaning (*P* < 0.05). The differences revealed that Dex showed excellent analgesic and sedative effects and could effectively reduce the incidence of complications after TURP, including cystospasm and nausea. In addition, it helped improve nursing satisfaction and patient prognosis.

## 1. Introduction

With the aggravation of population aging in China and the changes of people's dietary habits as well as lifestyles, the incidence of benign prostatic hyperplasia (BPH) is growing day by day [1, 2]. BPH is a common disease among elderly males, especially among those over 60. Relevant clinical reports indicate that the incidence of BPH among males over 60 is higher than 50%. Besides, the incidence grows with the increase of age. Furthermore, it reaches as high as 83% among males over 80 [3, 4]. Frequent micturition is the major symptom at early phase of BPH development. With the progress of the disease, some patients suffer from progressive dysuria. In addition, serious patients suffer from urinary retention due to severer obstruction [5].

The article "Analgesic Effects of Dexmedetomidine Combined with Spinal and Epidural Anesthesia Nursing on Prostate Hyperplasia Patients after Transurethral Resection of Prostate by Intelligent Algorithm-Based Magnetic Resonance Imaging" was published in 2022. Journal: Comput Math Methods Med.

At present, clinical therapeutic methods of prostate hyperplasia include drug treatment, microtraumatic operation, and surgical treatment. Transurethral resection of prostate (TURP) is the most frequently adopted method, which is honored as the “gold standard” for the treatment of BPH [6, 7]. Compared with open surgeries, TURP is featured with short operation time and significant therapeutic effects. It can effectively reduce hospitalization time and prognosis of patients [8]. However, most elderly patients suffer from complicated hypertension, coronary disease, diabetes, chronic obstructed lung diseases, and other chronic diseases because of the degeneration of each body function. As a result, patients show poor tolerance during surgery. In particular, pain after TURP affects the living quality and recovery rate of patients remarkably. Patients with severe pains even suffer from cystospasm [9, 10], which is induced by the injuries in urinary bladder areas during TURP and long postoperative catheter retention. Acute pain results in tension and anxiety among patients. Furthermore, it induces cardiovascular and cerebrovascular accidents and exacerbates patients' disease [11, 12]. Hence, it is indispensable to offer analgesic therapy to patients after TURP. Clinically, the common analgesic treatment methods include patient-controlled epidural analgesia (PCEA) and patient-controlled intravenous analgesia (PCIA) [13]. By PCEA, analgesia patients can control the injection dose of medical solution according to their pain levels. The side effects of opiates are reduced, and patients' analgesic needs can be met [14]. The drugs commonly adopted in CEA are local anesthetics and opiates, which show poor analgesic effects and cause nausea, emesis, drug dependence, and other side effects [15]. Dexmedetomidine (Dex) is a highly selective *α*2-adrenergic receptor agonist, which can act directly on peripheral *α*2 receptors, reduce the release of norepinephrine, and further show sedative and analgesic effects [16]. Chen et al. [17] applied Dex combined with ropivacaine in parturition analgesia successfully with excellent application effects.

The article "Analgesic Effects of Dexmedetomidine Combined with Spinal and Epidural Anesthesia Nursing on Prostate Hyperplasia Patients after Transurethral Resection of Prostate by Intelligent Algorithm-Based Magnetic Resonance Imaging" was published in 2022. Journal: Comput Math Methods Med.

In clinical practice, the main methods of assessing residual or recurrence after TURP include computed tomography (CT), magnetic resonance imaging (MRI), and ultrasound. MRI shows high resolution, and it can clearly display the internal structure of prostatic soft tissues. With the continuous development of imaging technology, MRI technology is applied in clinical practice more and more widely. In addition, the demand for measuring the size and position of prostates by MRI is gradually growing [18]. In previous clinical practice, doctors need to manually sketch prostates and then measure their size and location. In addition, artifacts and noises appear in original image due to various objective factors. As a result, there is the difference in the quality of original images. Hence, it takes a long time in the field of medical enhancement processing. It is now necessary to search for an efficient processing method. Deep learning focuses on the task analysis in a data-driven way and can intensively learn relevant model characteristics and data features from the massive data of specific problems automatically. Different from the hand-designed models displayed for specific problems, its learning process is essentially a procedure of solving an optimization problem. Hence, deep learning is widely applied in medical image processing [19].

To sum up, the present safety of anesthesia nursing for patients with BPH surgery was insufficient. The search for a more reliable anesthetic plan is a hot topic of the current research. Based on this, Mask R-CNN algorithm-based MRI image segmentation model was proposed in the research, and the model was utilized to investigate the analgesic effects of Dex with combined spinal and epidural anesthesia nursing on prostate hyperplasia patients after TURP. The investigation was expected to provide data support for the application of Dex with combined spinal and epidural anesthesia nursing in alleviating the postoperative pains of TURP patients.

## 2. Methods and Materials

### 2.1. Research Objects

In this research, a total of 184 patients receiving TURP in hospital between June 2018 and June 2020 were selected as the research objects. According to random number table method, all patients were divided into groups A, B, C, and D with 46 cases in each. This research had been approved by ethics committee of hospital. Besides, patients and their family members had been informed of the research and signed the informed consent forms.

*Inclusion criteria*. Patients were over 60 years old. Patients selected combined spinal and epidural anesthesia for the implementation of TURP. Patients utilized PCEA. Patients were graded at I and III by the American Society of Anesthesiologists (ASA) [20]. Patients showed no mental disorders. Patients did not suffer from severe cardiovascular and cerebrovascular diseases. Patients did not take analgesic and sedative drugs for long previously.

The article "Analgesic Effects of Dexmedetomidine Combined with Spinal and Epidural Anesthesia Nursing on Prostate Hyperplasia Patients after Transurethral Resection of Prostate by Intelligent Algorithm-Based Magnetic Resonance Imaging" was published in 2022. Journal: Comput Math Methods Med.

*Exclusion criteria*. Patients suffered from severe basic diseases. Patients were graded at III and above by ASA. Patients were allergic to the drugs adopted in the research. Patients showed poor compliance so that they could not be cooperative in the research.

### 2.2. Grouping Experiment

Patients in four groups were treated with 0.1% ropivacaine (hydrochloride ropivacaine injection with the dose of 100 mg/10 mL/each) as the analgesic drug solution, and all self-control analgesia devices PCEA were connected 10 minutes before the treatment.

In group A, patients were treated with 0.1% ropivacaine and 0.5 *μ*g/kg Dex. The total amount of configuration was 150 mL. Besides, the operation rate of analgesic pumps reached 3 mL/h with the amount of each press being 3 mL and the extreme amount being 10 mL. The locking time was 20 minutes.

In group B, patients were treated with 0.1% ropivacaine and 1 *μ*g/kg Dex. The total amount of configuration was 150 mL. Besides, the operation rate of analgesic pumps reached 3 mL/h with the amount of each press being 3 mL and the extreme amount being 10 mL. The locking time was 20 minutes.

In group C, patients were treated with 0.1% ropivacaine and 2 *μ*g/kg Dex. The total amount of configuration was 150 mL. Besides, the operation rate of analgesic pumps reached 3 mL/h with the amount of each press being 3 mL and the extreme amount being 10 mL. The locking time was 20 minutes.

Group D was the blank control group. All patients in this group were treated with 0.1% ropivacaine. The total amount of configuration was 150 mL. Besides, the operation rate of analgesic pumps reached 3 mL/h with the amount of each press being 3 mL and the extreme amount being 10 mL. The locking time was 20 minutes.

### 2.3. Anesthesia Methods

In the research, epidural anesthesia puncture kits were selected. After conventional sterilization, the third and fourth lumbar interstitial middle lines were selected as the puncture points. After the local infiltration and anesthesia by lidocaine, puncture was performed with 18G epidural puncture needles. The needles were pierced into epidural space slowly, and then, 25G spinal anesthesia needles were utilized. After the needle core was removed, cerebrospinal fluid flew out, which indicated successful puncture. After that, 0.67% 2 to 3 mL of ropivacaine was injected into subarachnoid space, and then, epidural catheters were retained. After ensuring that no blood or cerebrospinal fluid flew out by pumpback, catheters were fixed.

The article "Analgesic Effects of Dexmedetomidine Combined with Spinal and Epidural Anesthesia Nursing on Prostate Hyperplasia Patients after Transurethral Resection of Prostate by Intelligent Algorithm-Based Magnetic Resonance Imaging" was published in 2022. Journal: Comput Math Methods Med.

### 2.4. Imaging Examination Methods

In the research, 3.0T magnetic resonance scanner was utilized, body coils were adopted as radiofrequency emission coils, and the receiving coils were pelvic phased array coils for examination. The subjects were asked to take supine position. The superior border of symphysis pubis was at the center of coils, and cross-sectional scanning range covered patients' prostates and seminal vesicles. The scanning parameters included T1-weighted imaging at axial planes (layer thickness was 4 mm, layer spacing was 0.8 mm, matrix size was 512 × 512, and the number of excitation was 2.0), T2-weighted imaging (layer thickness was 4 mm, layer spacing was 0.8 mm, matrix size was 512 × 512, and the number of excitation was 2.0), and T1-weighted imaging at sagittal planes (layer thickness was 4 mm, layer spacing was 0.8 mm, matrix size was 512 × 512, and the number of excitation was 4.0).

The analysis of images was as follows. All MRI images were imported in dcm format and then saved in hard disks. Then, Mask R-CNN [21], U-net [22], and V-net [23] were adopted to segment the imported MRI images, and the segmentation effects were evaluated by two doctors with similar qualifications.

### 2.5. Mask R-CNN Algorithm

Mask R-CNN is composed mainly of feature extraction network, region proposal network, and networks heads, as shown in Figure 1 below. The feature extraction network of feature pyramid networks (FPN) extracts the features at the different levels from the input images, and then, the regions to be examined that contain segmentation targets are generated by region proposal network (RPN). After that, the image features of regions to be examined are acquired by the counterpropagation of ROI Align. Finally, the image features extracted by ROI Align are transmitted to network heads, and the segmentation results of modified target regions are acquired after classification, regression, and Mask operation. In the end, nonmaximum suppression (NMS) is adopted to extract the final segmentation results in target examination.

### 2.6. Postoperative Follow-Up Visits and Observation

In terms of postoperative follow-up visits, each of patients' indexes was observed 8 hours, 12 hours, 24 hours, and 48 hours after the operation, respectively, in the research, including pain visual analogue scale (VAS), sedation scores (Ramsay), patient-controlled epidural analgesia (PCEA) press numbers, incidence of cystospasm, nausea, emesis, pruritus, heart rate (HR), blood pressure (BP), oxygen saturation (SPO_2_), and nursing satisfaction.

In terms of VAS, patients' pain levels were assessed 8 hours, 12 hours, 24 hours, and 48 hours after the operation, respectively.  Table 1 shows pain grading below. VAS scores for pains ranged between 0 and 10 points. A higher score indicated severer pains for patients.

The article "Analgesic Effects of Dexmedetomidine Combined with Spinal and Epidural Anesthesia Nursing on Prostate Hyperplasia Patients after Transurethral Resection of Prostate by Intelligent Algorithm-Based Magnetic Resonance Imaging" was published in 2022. Journal: Comput Math Methods Med.

As for sedation scores (Ramsay), sedation scoring for patients was implemented 8 hours, 12 hours, 24 hours, and 48 hours after the operation, respectively. In sedation scoring system, level 1 (scored 1 point) showed patients' anxiety and dysphoria, level 2 (scored 2 points) indicated that patients could be cooperative and quiet, level 3 (scored 3 points) patients showed responses to all stimuli, level 4 (scored 4 points) demonstrated that patients responded quickly to knocking on glabella and other stimuli, level 5 (scored 5 points) revealed that patients responded slowly to knocking on glabella and other stimuli, and level 6 (scored 6 points) meant that patients did not respond to knocking on glabella and other stimuli.

Regarding nursing satisfaction, there were four levels of satisfaction, including high satisfaction, intermediate satisfaction, mild satisfaction, and high dissatisfaction. Nursing satisfaction consisted of high satisfaction, intermediate satisfaction, and mild satisfaction.

### 2.7. Algorithm Performance Evaluation Indexes

Dice similarity coefficient (DSC) is a common index of evaluating image segmentation effects, whose calculation equation is shown in equation (1) below.

(1) $$\begin{array}{c} \text{DSC}=\frac{2\left|C\cap D\right|}{\left|C\right|+\left|D\right|}. \end{array}$$

In equation (1), *C* referred to the target regions predicted by the algorithm and *D* denoted the standard target regions. A higher Dice value revealed better segmentation effects. In addition, the sensitivity, specificity, and positive predictive value (Ppv) of three algorithms were compared in the research. Equations (2)–(4) demonstrated the calculation methods of the above three values below.

(2) $$\begin{array}{c} \text{Sensitivity}=\frac{\text{TP}}{\text{TP}+\text{FN}}, \end{array}$$

(3) $$\begin{array}{c} \text{Specificity}=\frac{\text{TN}}{\text{TN}+\text{FP}}, \end{array}$$

(4) $$\begin{array}{c} \text{Ppv}=\frac{\text{TP}}{\text{TP}+\text{FP}}. \end{array}$$

In equations (2)–(4), TP referred to true positive value, TN denoted true negative value, FP represented forecast positive value, and FN stood for forecast negative value.

### 2.8. Statistical Analysis

In the research, data were processed by statistical product and service solutions (SPSS) 21.0. Measurement data were expressed by mean ± deviation ($\bar{x}\pm s$). Quantitative data with compound normal distribution were analyzed by variance, and qualitative data were tested by chi-square method. Besides, quantitative data and qualitative data without normal distribution were tested by nonparameters. *P* < 0.05 indicated that all differences showed statistical significance.

The article "Analgesic Effects of Dexmedetomidine Combined with Spinal and Epidural Anesthesia Nursing on Prostate Hyperplasia Patients after Transurethral Resection of Prostate by Intelligent Algorithm-Based Magnetic Resonance Imaging" was published in 2022. Journal: Comput Math Methods Med.

## 3. Results

### 3.1. Comparison of General Clinical Data on Patients in Four Groups

In the research, the general data on patients in four groups were collected and compared, and the results are displayed in Table 2 below. The differences in average age, weight, height, and operation time of patients in four groups all showed no statistical significance (*P* > 0.05), which further verified the feasibility of the research.

### 3.2. Performance Analysis of Three Algorithms

DSC value of Mask R-CNN algorithm was 0.623 ± 0.084, which was higher than that of U-net and V-net algorithms. In contrast, the sensitivity of Mask R-CNN algorithm was 67.33%, which was lower than that of U-net (71.21%) and V-net (72.33%) algorithms. The specificity of Mask R-CNN algorithm reached 98.61%, which was higher than that of U-net (94.22%) and V-net (93.17%) algorithms. The Ppv of Mask R-CNN algorithm amounted to 69.57%, which was higher than that of U-net (64.22%) and V-net (65.39%) algorithms. Besides, the average calculation time of Mask R-CNN algorithm was 129.16 ± 13.24 ms, which was higher than that of U-net and V-net algorithms.  Figure 2 shows the comparison of performance of three algorithms below.

Figure 3 shows the segmentation results of three algorithms below. According to Figure 3, the segmentation results of U-net and V-net algorithms displayed vague boundaries with many sawteeth. In contrast, the segmentation results of Mask R-CNN algorithm presented smooth boundaries and more accurate images.

### 3.3. Postoperative VAS Scores for Patients in Four Groups

VAS scores for group B 8 hours, 12 hours, 24 hours, and 48 hours after operation were 2.16 ± 0.33, 2.03 ± 0.38, 1.47 ± 0.41, and 0.85 ± 0.14, respectively, and those for group C were 1.76 ± 0.21, 1.65 ± 0.39, 1.26 ± 0.15, and 0.27 ± 0.15, respectively. Besides, VAS scores for groups B and C at different time periods were both obviously lower than that for group D, and the differences showed statistical significance (*P* < 0.05). In contrast, VAS scores for groups B and C at different time periods showed no obvious differences without statistical significance (*P* < 0.05).  Figure 4 demonstrates the comparison of VAS scores for four groups after operation below.

### 3.4. Sedation Scores for Patients in Four Groups after Operation

Ramsay scores for group B 8 hours, 12 hours, 24 hours, and 48 hours after operation were 1.42 ± 0.17, 0.93 ± 0.22, 0.85 ± 0.23, and 0.69 ± 0.17, respectively, and those for group C were 1.48 ± 0.16, 1.22 ± 0.24, 0.94 ± 0.21, and 0.81 ± 0.25, respectively. Ramsay scores for groups B and C at different time periods were both obviously higher than those of group D, and the differences showed statistical significance (*P* < 0.05). In contrast, Ramsay scores for groups A and D at different time periods showed no obvious differences without statistical significance (*P* > 0.05).  Figure 5 demonstrates the comparison of sedation scores for four groups after operation below.

The article "Analgesic Effects of Dexmedetomidine Combined with Spinal and Epidural Anesthesia Nursing on Prostate Hyperplasia Patients after Transurethral Resection of Prostate by Intelligent Algorithm-Based Magnetic Resonance Imaging" was published in 2022. Journal: Comput Math Methods Med.

### 3.5. Use of Other Analgesics among Patients in Four Groups

The use of other analgesics during follow-up visits among patients in four groups was as follows. During follow-up visits, the utilization of other analgesics among patients in four groups was 36.96% in group A, 13.04% in group B, 10.87% in group C, and 43.48% in group D, respectively. The results revealed that the utilization of other analgesics in groups B and C was obviously lower than that in group D, and the differences showed statistical significance (*P* < 0.05). In contrast, the utilization of other analgesics in groups A and D showed no obvious differences without statistical significance (*P* > 0.05).  Figure 6 displays the use of other analgesics among patients in four groups below.

### 3.6. Incidence of Cystospasm among Patients in Four Groups after Operation

During follow-up visits, the incidence of cystospasm in four groups was 26.67% in group A, 6.67% in group B, 2.17% in group C, and 36.67% in group D, respectively. The results showed that the incidence of cystospasm in groups B and C was obviously lower than that in group D, and the differences showed statistical significance (*P* < 0.05). In contrast, the incidence of cystospasm in groups A and D showed no obvious differences without statistical significance (*P* > 0.05).  Figure 7 presents the incidence of cystospasm among patients in four groups after operation below.

### 3.7. Nursing Satisfaction of Patients in Four Groups after Operation

During follow-up visits, the nursing satisfaction of patients in four groups was 26.09% in group A, 60.87% in group B, 73.91% in group C, and 23.91% in group D. According to the results, the nursing satisfaction in groups B and C was obviously higher than that in group D, and the differences showed statistical significance (*P* < 0.05). In contrast, the nursing satisfaction in groups A and D showed no obvious differences without statistical significance (*P* > 0.05).  Figure 8 displays the nursing satisfaction of patients in four groups after operation below.

## 4. Discussion

The incidence of BPH shows a growing trend year by year, and TURP is the main method of the clinical treatment of BPH. However, elderly patients can hardly endure pains after TURP due to their own chronic diseases. As a result, the prognosis of these patients was poor [24]. Clinically, analgesic drugs after TURP were opiates, such as fentanyl and morphine. Nevertheless, these drugs usually result in side effects, including nausea and emesis. Consequently, patients' living quality and nursing satisfaction were greatly reduced [25]. Based on the negative impacts of these drugs on the prognosis of patients, Mask R-CNN algorithm-based MRI image segmentation model was put forward in the research, and it was utilized to investigate the analgesic effects of Dex with combined spinal and epidural anesthesia nursing on prostate hyperplasia patients after TURP. In the research, U-net and V-net algorithms were introduced. In addition, DSC, sensitivity, specificity, Ppv, and operation time of three algorithms were compared. The results demonstrated that DSC value, specificity, and Ppv of Mask R-CNN algorithm were 0.623 ± 0.084, 98.61%, and 69.57%, respectively, all of which were higher than those of U-net and V-net algorithms. The results of the above comparison further verified the superiority of Mask R-CNN algorithm in image segmentation. Zhang et al. [26] adopted the deep learning of Mask R-CNN algorithm to offer a new method to the location and segmentation of MRI of breast lesions. Toufani et al. [27] utilized Mask R-CNN algorithm to segment the spinal cord cross-sectional area (SCCSA) of each section. The results revealed that the method showed high DSC, sensitivity, specificity, and accuracy, which was similar to the results of the research.

The article "Analgesic Effects of Dexmedetomidine Combined with Spinal and Epidural Anesthesia Nursing on Prostate Hyperplasia Patients after Transurethral Resection of Prostate by Intelligent Algorithm-Based Magnetic Resonance Imaging" was published in 2022. Journal: Comput Math Methods Med.

The patients were divided into group A (0.5 *μ*g/kg), group B (1 *μ*g/kg), group C (2 *μ*g/kg), and group D (0.1% of ropivacaine) according to different doses of Dex. In addition, VAS scores and Ramsay scores at different follow-up visit time, use of other analgesics, and incidence of postoperative cystospasm among patients in four groups were compared in the research. The results demonstrated that VAS scores for group B 8 hours, 12 hours, 24 hours, and 48 hours after operation were 2.16 ± 0.33, 2.03 ± 0.38, 1.47 ± 0.41, and 0.85 ± 0.14, respectively, and those for group C were 1.76 ± 0.21, 1.65 ± 0.39, 1.26 ± 0.15, and 0.27 ± 0.15, respectively. The scores for groups B and C were both obviously lower than those for group D, and the differences showed statistical significance (*P* < 0.05). Ropivacaine is a common amides local anesthesia drug, which is usually applied in short operations and is beneficial to the recovery of early activities after operation as well as the prevention of thrombus [28]. Dex plays significant roles in regulating immunization, reducing inflammatory reactions, and protecting nerves. At present, it is often applied in emergency operations, local and whole-body anesthesia, neurosurgery, pediatric surgical sedation, and bariatric surgical sedation. Zhang et al. [29] compared the auxiliary effects of Dex and sufentanil as local anesthetics on epidural parturition analgesia. The results showed that the analgesic effects and duration of the combined application of Dex and 0.1% of ropivacaine on the first labor of epidural analgesia were both better than those of sufentanil. The above outcome was similar to the result of the research. In addition, 2 *μ*g/kg dose of Dex showed better analgesic effects than 1 *μ*g/kg of Dex in the research.

The article "Analgesic Effects of Dexmedetomidine Combined with Spinal and Epidural Anesthesia Nursing on Prostate Hyperplasia Patients after Transurethral Resection of Prostate by Intelligent Algorithm-Based Magnetic Resonance Imaging" was published in 2022. Journal: Comput Math Methods Med.

Subramaniam et al. [30] compared the application of placebo combined with propofol and Dex in delirium after cardiac operation, and the results indicated that Dex reduced the incidence of delirium compared with placebo combined with propofol. In the research, Ramsay scores for groups B and C at different time periods were both obviously higher than those of group D (*P* < 0.05). The result was similar to that of the study conducted by Subramaniam et al. Furthermore, the incidence of cystospasm among patients in four groups during follow-up visits was compared in the research. The results demonstrated that the utilization of other analgesics in groups B and C was obviously lower than that in group D, and the differences showed statistical significance (*P* < 0.05). Cystospasm is a common complication after TURP and a significant factor causing postoperative acute pains. The main causes of the incidence of cystospasm include inadequate drainage and catheter stimulation. Cheng et al. [31] evaluated the therapeutic effects and safety of phloroglucinol combined with parecoxib in cystospasm after TURP. The results showed that the method effectively reduced the incidence of cystospasm after TURP with higher levels of effectiveness and safety compared with the utilization of phloroglucinol alone. The result was similar to that of the research. Finally, postoperative nursing satisfaction of patients in four groups was evaluated in the research. The results revealed that the nursing satisfaction in groups B and C was obviously higher than that in group D, and the differences showed statistical significance (*P* < 0.05). According to the results in the research, the adoption of Dex in postoperative analgesia could effectively enhance patients' nursing satisfaction and further verified the feasibility of the application of Dex in analgesia after TURP.

## 5. Conclusion

To analyze the investigation of analgesic effects of different doses of Dex combined with spinal and epidural anesthesia nursing after TURP by intelligent algorithm-based MRI, MRI image segmentation model of Mask R-CNN algorithm was proposed in the research, and then, the segmentation effects of Mask R-CNN, U-net, and V-net algorithms were compared and analyzed. Besides, 184 patients receiving TURP were selected as the research objects and divided into four groups based on random number table method. Each group was offered different doses of Dex, and then, VAS scores and Ramsay scores at different follow-up visit time, use of other analgesics, incidence of postoperative cystospasm, and nursing satisfaction of patients in four groups were compared. The results demonstrated that Dex showed excellent analgesic and sedative effects and could effectively reduce cystospasm, nausea, and other complications after TURP. In addition, it helped improve nursing satisfaction and patient prognosis. However, there were some limitations in the research. For example, follow-up visit time was short so that long-term effects of Dex could not be observed. In future experiments, sample size needed to be enlarged and hemodynamics changes should be further investigated. In general, the research provided data support for the clinical application of Dex combined with ropivacaine and the postoperative analgesia for TURP patients.

The article "Analgesic Effects of Dexmedetomidine Combined with Spinal and Epidural Anesthesia Nursing on Prostate Hyperplasia Patients after Transurethral Resection of Prostate by Intelligent Algorithm-Based Magnetic Resonance Imaging" was published in 2022. Journal: Comput Math Methods Med.

## Figures and Tables

**Figure 1:** Process of Mask R-CNN algorithm.

**Figure 2:** Analysis of performance of three algorithms. (a) DSC values; (b) sensitivity; (c) specificity; (d) Ppv; (e) operation time.

**Figure 3:** Segmentation results of three algorithms. A and B referred to two cases. (a–d) The image to be divided, the segmentation result of U-net algorithm, the segmentation result of V-net algorithm, and the segmentation result of Mask R-CNN algorithm, respectively.

**Figure 4:** Comparison of VAS scores for patients in four groups after operation. (a) Eight hours after operation; (b) 12 hours after operation; (c) 24 hours after operation; (d) 48 hours after operation. ∗ indicated that the comparison with group D demonstrated that the differences showed statistical significance (*P* < 0.05).

**Figure 5:** Comparison of sedation scores for patients in four groups after operation. (a) Eight hours and 12 hours after operation; (b) 24 hours and 48 hours after operation. ∗ indicated that the comparison with group D demonstrated that the differences showed statistical significance (*P* < 0.05).

**Figure 6:** Use of other analgesics among patients in four groups. ∗ indicated that the comparison with group D demonstrated that the differences showed statistical significance (*P* < 0.05).

The article "Analgesic Effects of Dexmedetomidine Combined with Spinal and Epidural Anesthesia Nursing on Prostate Hyperplasia Patients after Transurethral Resection of Prostate by Intelligent Algorithm-Based Magnetic Resonance Imaging" was published in 2022. Journal: Comput Math Methods Med.

**Figure 7:** Incidence of cystospasm among patients in four groups after operation. ∗ indicated that the comparison with group D demonstrated that the differences showed statistical significance (*P* < 0.05).

**Figure 8:** Nursing satisfaction of patients in four groups after operation. ∗ indicated that the comparison with group D demonstrated that the differences showed statistical significance (*P* < 0.05).

**Table 1:** Pain VAS.

Pain degree	Explanations
No pain	VAS score was 0.
Mild	VAS scores ranged between 1 and 3. Patients could endure mild pains, and sleep was not affected.
Moderate	VAS scores ranged between 4 and 6. Patients could endure moderate pains, and sleep was disturbed.
Severe	VAS scores ranged between 7 and 10. Patients could not endure severe pains, and sleep was disturbed and severely disrupted.

**Table 2:** Comparison of general clinical data on the patients in the four groups.

Pain degree	Group B	Group B	Group C	Group D
Age (years old)	68.45 ± 4.81	69.23 ± 5.28	68.62 ± 4.23	67.84 ± 5.11
Height (cm)	165.32 ± 11.42	164.77 ± 9.44	166.04 ± 9.86	165.51 ± 10.37
Weight (kg)	62.44 ± 8.05	63.16 ± 7.13	62.78 ± 5.48	63.22 ± 5.28
Operation time (minutes)	85.45 ± ±10.55	84.67 ± 4.88	86.16 ± 6.14	85.27 ± 6.09

## Data Availability

The data used to support the findings of this study are available from the corresponding author upon request.
